The article "lncRNA DLEU2 Accelerates Oral Cancer Progression via miR-30a-5p/RAP1B Axis to Regulate p38 MAPK Signaling Pathway" was published in 2022. Journal: Dis Markers.

# lncRNA DLEU2 Accelerates Oral Cancer Progression via miR-30a-5p/RAP1B Axis to Regulate p38 MAPK Signaling Pathway

**DOI:** 10.1155/2022/9310048

**Published:** 2022-10-12

**Authors:** Wenbo Zhang, Yanchun Wang, Pu Xu, Yongxiu Du, Weiwei Guan

**Affiliations:** ^1^Department of Periodontitis, Affiliated Haikou Hospital, Xiangya Medical School, Central South University, Hainan Provincial Stomatology Centre, Haikou, Hainan 570208, China; ^2^The First Outpatient Department of the Stomatological Hospital Affiliated to Kunming Medical University, Kunming 650031, China; ^3^Department of Oral Implantation, Affiliated Haikou Hospital, Xiangya Medical School, Central South University, Hainan Provincial Stomatology Centre, Haikou, Hainan 570208, China; ^4^Department of Oral Mucosal Disease, Affiliated Haikou Hospital, Xiangya Medical School, Central South University, Hainan Provincial Stomatology Centre, Haikou, Hainan 570208, China

## Abstract

**Background:**

Oral cancer (OC) is common cancer in the world. Long noncoding RNAs (lncRNAs) have been shown to be involved in cancer regulation, including oral cancer (OC). The aim of this study was to investigate the role of lncRNA deleted in lymphocytic leukemia 2 (DLEU2) in oral cancer.

**Method:**

The Gene Expression Omnibus database was used to analyze differentially expressed lncRNA/microRNA (miRNA, miR)/mRNA. The expression levels of *DLEU2*, miR-30a-5p, and *RAP1B* in OC cells were detected by RT-qPCR. Dual-luciferase was used to analyze the binding of lncRNA/miRNA/mRNA. Cell Counting Kit-8 was used to measure cell proliferation. Transwell assay was used to inspect cell migration and invasion abilities. Western blot was used to detect MAPK pathway-related protein levels.

**Result:**

Our research shows that, in contrast to miR-30a-5p, *DLEU2* or *RAP1B* was upregulated in OC cells, and high expression of DLEU2 or RAP1B was associated with poorer overall survival. Inhibiting the expression of DLEU2 slowed the proliferation and reduced the ability of migration and invasion of Tca8113 and CAL-27 cells. miR-30a-5p was predicted to interact with *DLEU2* or *RAP1B* by bioinformatics, and dual-luciferase analysis confirmed this interaction. Notably, si-*DLEU2* suppressed RAP1B expression and protein level, and after overexpression of *RAP1B* in OC cells, reversal of suppressed *DLEU2* expression was observed. Furthermore, the inhibitory effect of si-*DLEU2* on MAPK signaling was reversed by overexpression of *RAP1B*. Therefore, si-*DLEU2* regulates MAPK signaling through the miR-30a-5p/*RAP1B* axis and inhibits OC development.

**Conclusion:**

DLEU2 contributed to proliferation, migration and invasion via miR-30a-5p/RAP1B axis to regulate MAPK signaling pathway in OC cells.

The article "lncRNA DLEU2 Accelerates Oral Cancer Progression via miR-30a-5p/RAP1B Axis to Regulate p38 MAPK Signaling Pathway" was published in 2022. Journal: Dis Markers.

## 1. Introduction

Oral cancer (OC) is common cancer in the world [1, 2], and the current treatment of OC is usually surgery combined with radiotherapy and chemotherapy [3], but the mortality rate of OC is still high [4], which is due to the degree of tumor invasion and progression affecting the survival of patients with OC. Moreover, once lymph node metastasis occurs, the risk to patients' lives will rise dramatically [5]. Therefore, early detection of OC is very important. Therefore, OC tumor markers have important clinical value for identifying the mechanism of occurrence and metastasis of OC and finding new therapeutic methods.

Study have found that long noncoding RNAs (lncRNAs, >200 nt) do not encode proteins [6] but can directly participate in the regulation of gene expression [7] and can also interact with miRNAs as competing endogenous RNAs (ceRNAs) [8]. miRNAs play key roles in the posttranscriptional regulation of mRNAs by targeting their 3′ untranslated regions (UTRs), leading to mRNA degradation or translational repression [9]. In recent years, many studies have found that lncRNAs are involved in the occurrence and development of OC as ceRNAs [10–12]. As a known oncogene, lncRNA deleted in lymphocytic leukemia 2 (DLEU2) plays a role in promoting cancer development in most cancers [13, 14], but the molecular mechanism in OC has not yet been reported.

In recent years, alterations in signaling pathways involved in OC have been shown to be important factors affecting OC development [15, 16]. Among them, the canonical mitogen-activated protein kinase (MAPK) signaling pathway is considered to be involved in the growth and development of most cells [17, 18]. As an important member of MAPK, phosphorylation of p38 MAPK mediates the migration and growth of OC cells [19].

In this article, we sought to examine the expression and molecular mechanism of lncRNA DLEU2 in OC and to evaluate its impact on the biological behavior of 2 OC cell lines. Furthermore, we revealed a novel mechanism by which lncRNA DLEU2 regulates OC cell proliferation and distal migration through miR-30a-5p/member of RAS oncogene family (RAP1B)/MAPK signaling, which may provide new ideas for the discovery of OC therapeutic strategies.

## 2. Materials and Methods

### 2.1. Microarray Raw Data Analyses

Raw data are from National Center for Biotechnology Information Gene Expression Omnibus (GEO, https://www.ncbi.nlm.nih.gov/geo/). The expression profiles of lncRNA/mRNA in OC samples (GSE25099) were analyzed using GEO, which were divided into two groups: from 10 normal oral tissues (GSM616588-GSM616597) and 10 OC patient tissues (GSM616647-GSM616656). The expression profiles of miRNAs in samples (GSE98463) were divided into two groups: from 4 normal oral tissues (GSM2596879-GSM2596882) and 4 OC patient tissues (GSM2596874-GSM2596877). Differentially expressed lncRNAs/mRNAs/miRNAs were identified according to the following criteria: *P* < 0.05 and |fold change| ≥ 2. A heat map or volcano plot was constructed using differentially expressed lncRNA/mRNA/miRNA analysis results. KEGG pathway enrichment analyses were performed using the functional annotation tool of DAVID Bioinformatics Resources 6.8 (https://david.ncifcrf.gov/summary.jsp). The miRNA-lncRNA interactions between lncRNA and miRNA were predicted using starBase (https://starbase.sysu.edu.cn/index.php). Putative targets of miRNA-mRNA were predicted using TargetScan 7.2 (https://www.targetscan.org/vert_72/).

The article "lncRNA DLEU2 Accelerates Oral Cancer Progression via miR-30a-5p/RAP1B Axis to Regulate p38 MAPK Signaling Pathway" was published in 2022. Journal: Dis Markers.

### 2.2. Cell Lines and Culture and Transfection

Human oral cancer cell lines (CAL-27, Tca8113, and C4-2, 22RV1), normal oral keratinocytes (NOKs), and human embryonic kidney cells 293 (HEK 293T) were purchased from American Type Culture Collection (ATCC; VA, USA). All cells were maintained in DMEM medium (HyClone, UT, USA) with 10% fetal bovine serum (FBS; HyClone). RNAs was transfected into cells using Lipofectamine 3000 (Invitrogen; Thermo Fisher Scientific, Inc.).

### 2.3. Transient DLEU2 Silencing

si-DLEU2-1, si-DLEU2-2, si-DLEU2-3, and scrambled siRNA (si-NC) were designed and synthesized by Sigma-Aldrich. The siRNA sequences were as follows: si-DLEU2-1, 5′-GGTACTTCACTATAGTTTAdTdT-3′; si-DLEU2-2, 5′-GAATAACATCAATATGCAAdTdT-3′; si-DLEU2-3, 5′-GTATGAGAATATTATACTAdTdT′; and si-NC, 5′-TTCTCCGAACGTGTCACGdTdT-3′. After the above siRNAs were transfected into Tca8113 and CAL-27 cells, the cells were harvested 24 hours later. The inhibitory efficiency of the three si-DLEU2 was evaluated by RT-qPCR, and the siRNA with the best inhibitory efficiency will be used as a DLEU2 antagonist for subsequent research and analysis.

### 2.4. RNA Isolation and Quantitative RT-qPCR Analysis

Total RNA was extracted from cells using TRIzol (Invitrogen, MA, USA) according to the manufacturer's instructions. Real-time mRNA quantification for *DLEU2*, miR-30a-5p, *RAP1B*, *U6*, and 18sRNA was performed using SYBR Green qPCR SuperMix (Invitrogen) on a 7500 RT-qPCR System (Applied Biosystems, MA, USA). PCR experiments were carried out under the following conditions: 95°C for 10 min, 55°C for 2 min, and 72°C for 2 min, followed by 40 cycles of 95°C for 15 s and 60°C for 1 min. The primers for *DLEU2*, *RAP1B*, miR-30a-5p, 18sRNA (as internal normalization control for *DLEU2* and *RAP1B*), and U6 (as internal normalization control for miR-30a-5p) were as follows: *DLEU2* forward, 5′-TCCTTCCCTGGAAGAGCACA-3′, and *DLEU2* reverse, 5′-TTGGAGCTGCTATGCTTGTCA-3′; *RAP1B* forward, 5′-ACAGCGTGAGAGGTACTAGGT-3′, and *RAP1B* reverse, 5′-GTAAATTGCTCCGTTCCTGC-3′; miR-30a-5p forward, 5′-ACACTCCAGCTGGGTGTAAACATCCTCGAC-3′, and miR-30a-5p reverse, 5′-CTCAACTGGTGTCGTGGA-3′; 18sRNA forward, 5′-CCTGGATACCGCAGCTAGGA-3′, and 18sRNA reverse, 5′-GCGGCGCAATACGAATGCCCC-3′; and U6 forward, 5′-CTCGCTTCGGCAGCACA-3′, and U6 reverse, 5′-AACGCTTCACGAATTTGCGT-3′. Relative *DLEU2*, *RAP1B*, and miR-30a-5p expression levels were calculated using the 2^−*ΔΔ*Ct^ method [20]. All RT-PCR experiments were repeated three times.

The article "lncRNA DLEU2 Accelerates Oral Cancer Progression via miR-30a-5p/RAP1B Axis to Regulate p38 MAPK Signaling Pathway" was published in 2022. Journal: Dis Markers.

### 2.5. Cell Proliferation Rate

Cell Counting Kit-8 (CCK8) reagent (Solarbio; 10 *μ*L) was added to 96-well plates (containing Tca8113 and CAL-27 4 × 10^3^ cells) at 0, 24, 48, and 72 h, respectively. The absorbance was measured at 450 nm using an enzyme-labeled instrument (Thermo Fisher Scientific) after 60 min of incubation in the dark at 37°C.

### 2.6. Transwell Migration and Invasion Assays

The migration and invasion of Tca8113 and CAL-27 cells were determined using 24-well Transwell inserts (BD Biosciences). For the migration assay, the cells (0.5 × 10^5^) in serum-free medium were placed in the top chamber, whereas culture medium containing 10% FBS was added to the lower chamber. After incubating for 24 h, invasive cells were fixed using anhydrous ethanol for 30 min and stained with 0.1% crystal violet (Solarbio; 25°C) for 25 min. The cells were counted using a light microscope (Olympus Corporation) at ×200 magnification. For the invasion assay, inserts were first coated with Matrigel® (BD Biosciences) for 6 h at 37°C, then fixed, stained, and counted.

### 2.7. Dual-Luciferase Reporter Assay

The whole sequence of *DLEU2* or *RAP1B* 3′UTR was inserted into the psi-CHECK2 basic construct. We transfected HEK 293 T cells with a 0.5 *μ*g reporter construct and 50 nM miRNA mimic per well using Lipofectamine 3000. Following 4 h of transfection, the transfection medium was replaced with complete culture medium. Following 48 h of culture, the cells were lysed with passive lysis buffer (Promega), and luciferase activity was measured at 490 nm using the dual-luciferase reporter assay system (Promega). The ratio of firefly to *Renilla* luciferase activity was used to normalize firefly luciferase values.

### 2.8. Western Blotting

Tca8113 and CAL-27 cells were lysed using RIPA lysis buffer (Solarbio) and estimated using a BCA protein assay kit (Solarbio). Denatured proteins were resolved using 10% sodium dodecyl sulfate-polyacrylamide gel electrophoresis (SDS-PAGE, Solarbio), and protein bands were transferred to a polyvinylidene fluoride membrane, blocked with 5% bovine serum albumin (Solarbio), and incubated overnight (4°C) with RAP1B (1 : 500; ab154756, Abcam, Cambridge, UK), p38 (1 : 1000; ab170099, Abcam), and p-p38 (1 : 1000; ab178867, Abcam) primary antibodies. Thereafter, the sections were rinsed with TBST buffer (Solarbio; containing 0.05% Tween 20) twice for 15 min and incubated with goat anti-rabbit antibody (1 : 20,000, ab205718; Abcam) for 2 h at 25°C. Anti-GAPDH antibody (1 : 5,000, ab181602; Abcam) was used as a loading control. Proteins were visualized using Immobilon Western Chemiluminescent HRP Substrate (Millipore). Chemiluminescence signal acquisition was performed using an X-ray film (Kodak).

The article "lncRNA DLEU2 Accelerates Oral Cancer Progression via miR-30a-5p/RAP1B Axis to Regulate p38 MAPK Signaling Pathway" was published in 2022. Journal: Dis Markers.

### 2.9. Statistical Analysis

Statistical analysis was performed using GraphPad Prism software (v8.3.0), and data were expressed as mean ± SD. To determine whether there was an overall statistically significant difference, a one-way ANOVA was performed with a Bonferroni post hoc test before Student's *t*-test was performed to analyze the difference between any two groups. It was considered statistically significant if *P* > 0.05.

## 3. Results

### 3.1. DLEU2 Is Upregulated in OC Cells

Analysis of the results of OC patients and normal subjects based on lncRNA microarray data identified 20 differentially expressed transcripts of lncRNAs, including 15 upregulated and 5 downregulated (Figure 1(a)). Among them, DLEU2, as a known oncogene, expression was upregulated in the dataset and has not yet been studied on the molecular mechanism in OC. Furthermore, based on RT-qPCR assays, DLEU2 expression was significantly upregulated in 4 OC cells (CAL-27, FaDu, HSC-2, and Tca8113) (Figure 1(b)). Therefore, we have reason to believe that DLEU2 may be closely related to the development of OC. Notably, DLEU2 was most expressed in Tca8113 and CAL-27 cells, so these two cell lines were selected to explore the functional role of DLEU2 in OC. RT-qPCR results showed that after transfecting the synthesized three kinds of siRNA-DLEU2 into Tca8113 and CAL-27 cells, siRNA-DLEU2-1 was found to have the best inhibitory effect. We used it as an antagonist of DLEU2 to study the molecular mechanism (Figure 1(c)). The results of CCK8 and Transwell showed that inhibiting the expression of DLEU2 slowed the proliferation of Tca8113 and CAL-27 cells and reduced the ability of migration and invasion (Figures 1(d)–1(g)). Furthermore, by RT-qPCR analysis, we observed that DLEU2 was mainly distributed in the cytoplasm of cells (Figure 1(h)), so the effect of DLEU2 on OC might be achieved through a ceRNA mechanism.

### 3.2. DLEU2 Directly Targets miR-30a-5p

According to the miRNA microarray data analysis results, using 4 OCs and 4 normal oral tissues, 209 differentially expressed hsa-miRNAs were identified, of which 88 were upregulated and 121 miRNAs including miR-30a-5p were downregulated (Figure 2(a)). Combined with the analysis of starBase database and miRNA microarray (Figure 2(b)), we observed that 3 miRNAs intersected, and miR-30a-5p was confirmed to be downregulated in OC [21], so we screened it as a potential target of DLEU2. The results showed that miR-30a-5p was downregulated in OC cells (Figure 2(c)), and inhibiting the expression of DLEU2 could increase the expression of miR-30a-5p (Figure 2(d)). The starBase database predicts that DLEU2 has a binding site for miR-30a-5p (Figure 2(e)); subsequent dual-luciferase experiments confirmed that DLEU2 directly targets miR-30a-5p (Figure 2(f)). Here, we can confirm that DLEU2 can sponge miR-30a-5p to regulate OC development.

The article "lncRNA DLEU2 Accelerates Oral Cancer Progression via miR-30a-5p/RAP1B Axis to Regulate p38 MAPK Signaling Pathway" was published in 2022. Journal: Dis Markers.

### 3.3. RAP1B Directly Targets miR-30a-5p

According to the mRNA microarray data analysis results, a total of 1496 upregulated mRNAs including RAP1B were identified (Figure 3(a)). KEGG can analyze and predict that different mRNAs affect different signaling pathways. We found that the classical MAPK involved in cell growth and development is one of the key signaling pathways that affect the progression of OC (Figure 3(b)), and 44 mRNAs are predicted to be involved. Combined with the 4117 potential target genes of miR-30a-5p predicted by the starBase database, we observed that 8 mRNAs intersected (Figure 3(c)). The study has confirmed that RAP1B is upregulated in OC [22]; therefore, we screened the RAP1B gene as a potential target for validation. The QRT-PCR results showed that RAP1B was highly expressed in OC cells (Figure 3(d)). The TargetScan database predicts that RAP1B has a binding site for miR-30a-5p (Figure 3(e)); subsequent dual-luciferase assays confirmed that RAP1B directly targets miR-30a-5p (Figure 3(f)). After transfection of si-DLEU2, RAP1B expression was downregulated in Tca8113 and CAL-27 cells (Figure 3(g)).

### 3.4. DLEU2 Is Positively Correlated with RAP1B

To confirm the association between DLEU2 and RAP1B, we constructed a RAP1B overexpression plasmid (ov-RAP1B). The QRT-PCR and western blot results indicated that the gene or protein levels of RAP1B was upregulated in ov-RAP1B-transfected Tca8113 and CAL-27 cells, confirming the effectiveness of the RAP1B overexpression plasmid (Figures 3(h) and 3(i)). After cotransfection with the addition of si-DLEU2, the inhibition of DLEU2 expression was reversed by ov-RAP1B (Figure 3(j)). Thus, miR-30a-5p directly targets DLEU2 and RAP1B, and DLEU2 positively correlates with RAP1B.

The article "lncRNA DLEU2 Accelerates Oral Cancer Progression via miR-30a-5p/RAP1B Axis to Regulate p38 MAPK Signaling Pathway" was published in 2022. Journal: Dis Markers.

### 3.5. The DLEU2/miR-30a-5p/RAP1B Axis Affects OC Development through MAPK Signaling

The above results suggest that MAPK is one of the key signaling pathways affecting OC development, and p38 MAPK is the core protein of MAPK. Based on western blot results, we found that knockdown of DLEU2 significantly reduced p-p38 MAPK protein levels in Tca8113 and CAL-27 cells (Figure 4(a)). However, the presence of ov-RAP1B reversed the effect of si-DLEU2 (Figure 4(b)). In addition, the results of cell function experiments showed that si-DLEU2 inhibited the proliferation of Tca8113 and CAL-27 cells (Figures 4(c) and 4(d)), and the effects of reducing migration and invasion ability (Figures 4(e) and 4(f)) were also reversed by ov-RAP1B. In conclusion, the DLEU2 sponge adsorbs miR-30a-5p and regulates the transcription and translation of RAP1B, thereby affecting downstream MAPK signaling and intervening in OC development.

## 4. Discussion

Our goal was to identify a novel lncRNA as a potential therapeutic target for OC therapy; therefore, a comprehensive understanding of the regulatory mechanisms of lncRNAs may help to develop new and promising therapeutic strategies for OC. Previous reports indicated that lncRNAs are important players in the development of OC [23]. For example, Zhang et al. [24] found that the lncRNA LINC01296 promoted the development of oral squamous cell carcinoma by binding to SRSF1. Lu et al. [25] demonstrated that lncRNA HOTAIR inhibited cancer stemness and metastasis in oral cancer stem cells. In our study, the oncogenic roles of DLEU2 and RAP1B in OC and the tumor suppressor role of miR-30a-5p were first determined. Mechanistically, we found that DLEU2 sponges adsorb miR-30a-5p, RAP1B is a target of miR-30a-5p, and DLEU2 is upregulated synergistically with RAP1B in OC progression. In addition, si-DLEU2 also inhibited the p38 MAPK pathway. MAPK family members mediate a variety of cellular behaviors in response to extracellular stimuli [26]. As one of the major members of MAPKs, p38 MAPKs function in a cell environment-specific and cell type-specific manner to integrate signals affecting proliferation and migration [18]. Taken together, our results suggest that the DLEU2/miR-30a-5p/RAP1B axis can regulate the progression of OC through the p38 MAPK pathway, providing a new therapeutic strategy for OC.

In various cancers, DLEU2 plays a promoting regulatory role in a variety of cancers. For example, He et al. found that DLEU2 promotes cervical cancer progression [27] and promotes the proliferation and invasive capacity of colorectal cancer cells [28]. Likewise, our results showed that DLEU2 was upregulated in OC cells, its high expression significantly shortened the disease-free survival of OC patients, and si-DLEU2 inhibited OC cell proliferation, migration, and invasion by reducing the phosphorylation of p38 MAPK. It is suggested that DLEU2, as an oncogene, will block the development of OC when its expression is suppressed. In addition, DLEU2, as a ceRNA, plays a role in phagocytosing miRNAs in cancer. For example, Wu et al. found that DLEU2 accelerated tumorigenesis and invasion of non-small-cell lung cancer by sponging miR-30a-5p [29]. Li et al. [30] found that DLEU2 promotes gastric cancer progression through sponge adsorption of miR-23b-3p. In this study, inhibiting the expression of DLEU2 promoted the expression of miR-30a-5p in OC cells, so that the transcription and translation of RAP1B directly bound to miR-30a-5p were also simultaneously degraded. This result indicates that miR-30a-5p as a tumor suppressor gene was confirmed in this study, which is consistent with the previous studies on the role of miR-30a-5p in suppressing cancer such as breast cancer [31] and lung adenocarcinoma [32].

The article "lncRNA DLEU2 Accelerates Oral Cancer Progression via miR-30a-5p/RAP1B Axis to Regulate p38 MAPK Signaling Pathway" was published in 2022. Journal: Dis Markers.

The bioinformatics database predicted that miR-30a-5p targets the 3′UTR of RAP1B, and we confirmed its targeting mechanism by dual-luciferase reporter gene experiments. Furthermore, in OC cells, RAP1B expression was negatively correlated with miR-30a-5p expression. Notably, our study shows that RAP1B promotes OC progression. Furthermore, in the ceRNA axis, DLEU2 was coordinated upregulated with RAP1B, a target gene of miR-30a-5p, in OC cells, and DLEU2 decreased the expression of RAP1B, whereas overexpression of RAP1B reversed si-DLEU2-mediated degradation of p38 MAPK phosphorylation. These results suggest that si-DLEU2 exerts a tumor suppressor effect through the interaction with miR-30a-5p and RAP1B. Furthermore, the tumor suppressor effect of RAP1B on OC is consistent with its role in other cancers such as thyroid cancer [33] and colorectal cancer [34].

The MAPK pathway directly regulates OC development [35, 36]. In the present study, when the phosphorylation level of p38 MAPK was decreased, the proliferation inhibition, migration, and invasion abilities of OC cells were decreased. si-DLEU2 inhibited OC cell growth and decreased p38 MAPK phosphorylation levels. Excessive RAP1B promotes cancer cell development, elevates p38 MAPK phosphorylation levels, and reverses the effects of si-DLEU2 on OC cells. Therefore, the DLEU2-miR-30a-5p-RAP1B axis controls the p38 MAPK signaling pathway, thereby regulating OC progression.

In conclusion, this study confirms that DLEU2 is a potential therapeutic target and provides more directions and theoretical basis for the treatment of OC.

## Figures and Tables

**Figure 1:** DLEU2 is a new potential target that promotes oral cancer development. (a) Hierarchical clustering heat map shows differentially expressed lncRNA including DLEU2 between the oral cancer and control groups. (b) Relative expression of DLEU2 in RWPE-2 and four oral cancer cell lines (C4-2, 22RV1, Tca8113, and CAL-27). (c) RT-qPCR analysis of the inhibition efficiency of 3 si-DLEU2 in Tca8113 and CAL-27 cells. (d, e) CCK8 analysis of the effect of si-DLEU2 on the proliferation rate of Tca8113 (d) and CAL-27 (e) cells. (f, g) Transwell analysis of the effects of si-DLEU2 on migration and invasion of Tca8113 (f) and CAL-27 (g) cells. (h) RT-qPCR analysis of DLEU2 localization in Tca8113 and CAL-27 cells. ^∗^*P* < 0.05.

The article "lncRNA DLEU2 Accelerates Oral Cancer Progression via miR-30a-5p/RAP1B Axis to Regulate p38 MAPK Signaling Pathway" was published in 2022. Journal: Dis Markers.

**Figure 2:** DLEU2 sponge adsorbs miR-30a-5p. (a) Hierarchical clustering heat map shows differentially expressed miRNA between the oral cancer and control groups. (b) The miRNA chip and the starBase database were combined to analyze the potential miRNAs that bind to DLEU2. (c) Relative expression of miR-30a-5p in RWPE-2 and four oral cancer cell lines (C4-2, 22RV1, Tca8113, and CAL-27). (d) RT-qPCR analysis of the effect of si-DLEU2 on the expression of miR-30a-5p in Tca8113 and CAL-27 cells. (e) The starBase database predicts the binding sites of DLEU2 and miR-30a-5p. (f) Dual-luciferase assay analysis of the binding of DLEU2 to miR-30a-5p. ^∗^*P* < 0.05.

**Figure 3:** RAP1B targets miR-30a-5p and reverses the effects of si-DLEU2 in Tca8113 and CAL-27 cells. (a) Scatter plot shows differentially expressed mRNAs between the oral cancer and control groups. (b) KEGG pathway enrichment analysis. (c) The key mRNAs affecting the MAPK signaling pathway were combined with putative target genes of miR-30a-5p in the starBase database to screen for suitable mRNAs. (d) Relative expression of DLEU2 in RWPE-2 and four oral cancer cell lines (C4-2, 22RV1, Tca8113, and CAL-27). (e) The TargetScan database predicts the binding sites of miR-30a-5p and RAP1B. (f) Dual-luciferase assay analysis of the binding of RAP1B to miR-30a-5p. (g) RT-qPCR analysis of the effect of si-DLEU2 on the expression of RAP1B in Tca8113 and CAL-27 cells. (h) RT-qPCR verified the validity of overexpressing RAP1B plasmid. (i) Western blot verified the validity of overexpressing RAP1B plasmid. (j) RT-qPCR analysis of the reversal of DLEU2 expression by overexpressing RAP1B on si-DLEU2. ^∗^*P* < 0.05.

**Figure 4:** si-DLEU2 suppresses oral cancer cell growth via the MAPK pathway. (a) Western blot analysis of si-DLEU2-mediated protein levels of RAP1B, p38, and p-p38. (b) Western blot analysis of si-DLEU2-/ov-RAP1B-mediated protein levels of RAP1B, p38, and p-p38. (c, d) CCK8 analysis of the effect of si-DLEU2/ov-RAP1B coaction on the proliferation rate of Tca8113 (c) and CAL-27 (d) cells. (e, f) Transwell analysis of the effect of si-DLEU2/ov-RAP1B coaction on migration and invasion of Tca8113 (e) and CAL-27 (f) cells. ^∗^*P* < 0.05.

The article "lncRNA DLEU2 Accelerates Oral Cancer Progression via miR-30a-5p/RAP1B Axis to Regulate p38 MAPK Signaling Pathway" was published in 2022. Journal: Dis Markers.

## Data Availability

The data used to support the findings of this study are included within the article.

## Abbreviations

OC: Oral cancer
lncRNA: Long noncoding RNA
miRNA, miR: microRNA
ceRNAs: Competing endogenous RNAs
UTR: Untranslated region
MAPK: Mitogen-activated protein kinase
GEO: Gene Expression Omnibus
NOKs: Normal oral keratinocytes
DLEU2: Deleted in lymphocytic leukemia 2
RAP1B: Member of RAS oncogene family.

## References

[1] Chattopadhyay I., Verma M., Panda M. (2019). Role of oral microbiome signatures in diagnosis and prognosis of oral cancer. *Technology in Cancer Research & Treatment*.

[2] Wong T., Wiesenfeld D. (2018). Oral cancer. *Australian Dental Journal*.

[3] Levi L. E., Lalla R. V. (2018). Dental treatment planning for the patient with oral cancer. *Dental Clinics of North America*.

[4] Kane G., Petrosyan V., Ameerally P. (2019). Oral cancer treatment through the ages: part 1. *Journal of Oral and Maxillofacial Surgery*.

[5] Nagao T., Warnakulasuriya S. (2020). Screening for oral cancer: future prospects, research and policy development for Asia. *Oral Oncology*.

[6] Jathar S., Kumar V., Srivastava J., Tripathi V. (2017). Technological developments in lncRNA biology. *Advances in Experimental Medicine and Biology*.

[7] Ferre F., Colantoni A., Helmer-Citterich M. (2016). Revealing protein-lncRNA interaction. *Briefings in Bioinformatics*.

[8] Paraskevopoulou M. D., Hatzigeorgiou A. G. (2016). Analyzing MiRNA-LncRNA interactions. *Methods in Molecular Biology*.

[9] Afonso-Grunz F., Muller S. (2015). Principles of miRNA-mRNA interactions: beyond sequence complementarity. *Cellular and Molecular Life Sciences*.

[10] Fang X., Tang Z., Zhang H., Quan H. (2020). Long non-coding RNA DNM3OS/miR-204-5p/HIP1 axis modulates oral cancer cell viability and migration. *Journal of Oral Pathology & Medicine*.

[11] Zhou R. S., Zhang E. X., Sun Q. F. (2019). Integrated analysis of lncRNA-miRNA-mRNA ceRNA network in squamous cell carcinoma of tongue. *BMC Cancer*.

[12] Fang Z., Zhao J., Xie W., Sun Q., Wang H., Qiao B. (2017). LncRNA UCA1 promotes proliferation and cisplatin resistance of oral squamous cell carcinoma by sunppressing miR-184 expression. *Cancer Medicine*.

[13] Dong P., Xiong Y., Konno Y. (2021). Long non-coding RNA DLEU2 drives EMT and glycolysis in endometrial cancer through HK2 by competitively binding with miR-455 and by modulating the EZH2/miR-181a pathway. *Journal of Experimental & Clinical Cancer Research*.

The article "lncRNA DLEU2 Accelerates Oral Cancer Progression via miR-30a-5p/RAP1B Axis to Regulate p38 MAPK Signaling Pathway" was published in 2022. Journal: Dis Markers.

[14] Lu T., Wang R., Cai H., Cui Y. (2020). Long non-coding RNA DLEU2 promotes the progression of esophageal cancer through miR-30e-5p/E2F7 axis. *Biomedicine & Pharmacotherapy*.

[15] Nigam K., Srivastav R. K. (2021). Notch signaling in oral pre-cancer and oral cancer. *Medical Oncology*.

[16] Peng Q. S., Cheng Y. N., Zhang W. B., Fan H., Mao Q. H., Xu P. (2020). circRNA_0000140 suppresses oral squamous cell carcinoma growth and metastasis by targeting miR-31 to inhibit Hippo signaling pathway. *Cell Death & Disease*.

[17] Bharath Kumar V., Lin J. T., Mahalakshmi B. (2021). Platyphyllenone exerts anti-metastatic effects on human oral cancer cells by modulating cathepsin L expression, MAPK pathway and epithelial-mesenchymal transition. *International Journal of Molecular Sciences*.

[18] Wagner E. F., Nebreda A. R. (2009). Signal integration by JNK and p38 MAPK pathways in cancer development. *Nature Reviews. Cancer*.

[19] Kumar V. B., Lin S. H., Mahalakshmi B. (2020). Sodium Danshensu inhibits oral cancer cell migration and invasion by modulating p38 signaling pathway. *Frontiers in Endocrinology*.

[20] Livak K. J., Schmittgen T. D. (2001). Analysis of relative gene expression data using real-time quantitative PCR and the 2(-delta delta C(T)) method. *Methods*.

[21] Ruan P., Tao Z., Tan A. (2018). Low expression of miR-30a-5p induced the proliferation and invasion of oral cancer via promoting the expression of FAP. *Bioscience Reports*.

[22] Mitra R. S., Zhang Z., Henson B. S., Kurnit D. M., Carey T. E., D'Silva N. J. (2003). Rap1A and rap1B ras-family proteins are prominently expressed in the nucleus of squamous carcinomas: nuclear translocation of GTP-bound active form. *Oncogene*.

[23] Huang F., Xin C., Lei K., Bai H., Li J., Chen Q. (2020). Noncoding RNAs in oral premalignant disorders and oral squamous cell carcinoma. *Cellular Oncology (Dordrecht)*.

[24] Zhang Y., Wang A., Zhang X., Wang X., Zhang J., Ma J. (2021). lncRNA LINC01296 promotes oral squamous cell carcinoma development by binding with SRSF1. *BioMed Research International*.

[25] Lu M. Y., Liao Y. W., Chen P. Y. (2017). Targeting LncRNA HOTAIR suppresses cancer stemness and metastasis in oral carcinomas stem cells through modulation of EMT. *Oncotarget*.

[26] El Rawas R., Amaral I. M., Hofer A. (2020). Is p38 MAPK associated to drugs of abuse-induced abnormal behaviors?. *International Journal of Molecular Sciences*.

[27] He M., Wang Y., Cai J. (2021). LncRNA DLEU2 promotes cervical cancer cell proliferation by regulating cell cycle and NOTCH pathway. *Experimental Cell Research*.

[28] He X., Yu B., Kuang G. (2021). Long noncoding RNA DLEU2 affects the proliferative and invasive ability of colorectal cancer cells. *Journal of Cancer*.

The article "lncRNA DLEU2 Accelerates Oral Cancer Progression via miR-30a-5p/RAP1B Axis to Regulate p38 MAPK Signaling Pathway" was published in 2022. Journal: Dis Markers.

[29] Wu W., Zhao Y., Gao E. (2020). LncRNA DLEU2 accelerates the tumorigenesis and invasion of non-small cell lung cancer by sponging miR-30a-5p. *Journal of Cellular and Molecular Medicine*.

[30] Li G., Zhang Z., Chen Z., Liu B., Wu H. (2021). LncRNA DLEU2 is activated by STAT1 and induces gastric cancer development via targeting miR-23b-3p/NOTCH2 axis and Notch signaling pathway. *Life Sciences*.

[31] Xiong J., Wei B., Ye Q., Liu W. (2019). MiR-30a-5p/UBE3C axis regulates breast cancer cell proliferation and migration. *Biochemical and Biophysical Research Communications*.

[32] Chen S., Zhu X., Zheng J., Xu T., Xu Y., Chen F. (2021). miR-30a-5p regulates viability, migration, and invasion of lung adenocarcinoma cells via targeting ECT2. *Computational and Mathematical Methods in Medicine*.

[33] Wang P., Gu J., Wang K., Shang J., Wang W. (2019). miR-206 inhibits thyroid cancer proliferation and invasion by targeting RAP1B. *Journal of Cellular Biochemistry*.

[34] Zhou Z., Xu H., Duan Y., Liu B. (2020). MicroRNA-101 suppresses colorectal cancer progression by negative regulation of Rap1b. *Oncology Letters*.

[35] Li Z., Liu F. Y., Kirkwood K. L. (2020). The p38/MKP-1 signaling axis in oral cancer: impact of tumor-associated macrophages. *Oral Oncology*.

[36] Asoudeh-Fard A., Barzegari A., Dehnad A., Bastani S., Golchin A., Omidi Y. (2017). Lactobacillus plantarum induces apoptosis in oral cancer KB cells through upregulation of PTEN and downregulation of MAPK signalling pathways. *BioImpacts: BI*.

